RETRACTED

# Diagnostic Value of Multislice Spiral CT Cardiothoracic Combined with Angiography in Acute Chest Pain

**DOI:** 10.1155/2021/5549971

**Published:** 2021-02-20

**Authors:** Yinggan Du, Zetian Yang

**Affiliations:** ^1^Jinhua Municipal Central Hospital, Jinhua Hospital of Zhejiang University, Jinhua, Zhejiang 321000, China; ^2^Wuhan University, Wuhan, Hubei 430072, China; ^3^Zhongnan Hospital of Wuhan University, Wuhan, Hubei 430071, China

## Abstract

Acute chest pain is a common clinical emergency condition with a variety of causes, including acute coronary syndrome, pulmonary embolism, aortic coarctation, and pneumothorax. It is essential for emergency physicians to quickly and accurately understand the cause of acute chest pain. 64-slice spiral CT combined cardiothoracic angiography is an accurate and rapid way to diagnose and differentiate the cause of acute chest pain. 64-slice combined cardiothoracic angiography can accurately and rapidly display the thoracic aorta, both pulmonary arteries, the main trunk of the coronary artery and its major branches, and also provide a comprehensive view of both lungs and mediastinum, which is an effective test for the diagnosis and differential diagnosis of acute chest pain. Based on this, this study further investigated the value of 64-slice spiral CT triplex examination in the diagnosis of acute chest pain. The results showed that 64-slice spiral CT has the advantages of fast scanning speed, high resolution, and advanced postprocessing technology, and combined cardiothoracic angiography can quickly and accurately help emergency physicians analyze the cause of acute chest pain, which plays a very important role in formulating the correct treatment plan in a timely manner. At the same time, with the continuous development of CT technology, the temporal and spatial resolution has improved the quality of CT images, giving us more options to reduce the effective radiation dose and reduce the total amount of contrast, making the 64-row spiral CT cardiothoracic imaging more perfect.

## 1. Introduction

Acute chest pain is considered to be one of the most common causes of emergency care in adult patients [1]. One-stop imaging of the chest pain triad is feasible for use in the evaluation of patients in the emergency department for the etiology of acute chest pain [2]. However, only a small proportion of patients with acute chest pain have undergone this test, and one of the main reasons preventing the one-stop test from becoming a routine diagnostic test is the issue of radiation dose [3]. Therefore, we analyzed various techniques that can reduce the radiation dose in the one-stop examination [4–10]. Appropriate application of these techniques can significantly reduce the radiation dose, and patients with acute chest pain can have less radiation damage during the one-stop examination. Therefore, the differential diagnosis between acute coronary syndrome, pulmonary embolism, and the acute aortic syndrome is necessary for patients with acute chest pain. The differential diagnosis between acute coronary syndrome, pulmonary embolism, and the acute aortic syndrome is very easy for patients with acute chest pain with high-risk factors because the disease has typical clinical symptoms or laboratory tests. For example, significant electrocardiographic changes, the elevation of serum cardiac enzymes, and typical symptoms of angina pectoris can be diagnostic of the acute coronary syndrome [11]. A positive dimer test in pulmonary artery embolism and aortic coarctation often presents with significant changes in blood pressure, and symptoms such as severe sudden chest pain are often seen in patients with aortic coarctation; therefore, American College of Radiology standards state that electrocardiography and serum cardiac enzymes should be their preferred tests. However, in patients with moderate risk factors, the differential diagnosis is difficult due to the similarity of their symptoms and the lack of specificity of each disease presentation [12]. In addition, the various tests can be expensive and take a long time to perform.

RETRACTED

Traditionally, each examination mainly diagnosed one disease, e. g., coronary artery examination mainly provided information on coronary arteries, aortic examination mainly provided information on aortic disease, etc. [13–16]. However, with the development of multiatrial spiral, the tube ball rotation time is decreasing, the scan time is getting faster, and the rapid development of techniques such as cardiac gating makes it possible to evaluate coronary artery, aorta, and pulmonary artery simultaneously by one examination, and this technique which is called chest pain triple one-stop imaging examination can reduce the number of single examinations used to evaluate coronary artery disease, aortic disease, and pulmonary artery disease, as Figure 1 shows. Derived from cardiac gated coronary artery examination [17], the difference compared to the coronary artery is the longer scan range, usually from the thoracic inlet to the level of the diaphragm. Using a conventional retrospective ECG gated scan, data from all phases of several cardiac cycles need to be acquired in the breath-hold state and then the best phase is selected for data reconstruction, which has a lower pitch, usually and can be used in the emergency department to assess the etiology of acute chest pain and has potential applications for early diagnosis [18]. The application was evaluated in patients with acute chest pain with low to moderate risk factors, and its negative predictive value was reached. The advantage of the multirow spiral is that it allows rapid assessment of the main etiology of acute chest pain and has a high negative predictive value [19]. In addition to its diagnostic feasibility, the test has other advantages, such as the ability to reduce the number of diagnostic tests, the time of the patient′s examination, and the cost of medical tests [20]. It provides a cost-effective modality for patients presenting to the emergency department with acute chest pain [21]. The test is able to make a diagnosis of noncoronary origin, which accounts for approximately the proportion of patients with acute chest pain in the emergency department, and it can avoid additional tests for the diagnosis of cardiac disease in patients who do not experience serious side effects during days of follow-up [22–25]. Multirow spiral is considered to have the potential to improve the diagnosis of acute chest pain in patients with low to moderate risk factors [26].

RETRACTED

Acute chest pain is a common clinical emergency symptom with a variety of causes, including acute coronary syndrome, pulmonary embolism, aortic coarctation, pneumothorax, etc. It is crucial for emergency physicians to quickly and accurately understand the cause of acute chest pain. 64-slice combined cardiothoracic angiography can accurately and rapidly display the thoracic aorta, both pulmonary arteries, the main trunk of the coronary arteries and their major branches, and also provide a comprehensive picture of the two lungs and mediastinum, which is an effective examination method for the diagnosis and differential diagnosis of the cause of acute chest pain. In this paper, 64-row spiral CT cardiothoracic combined angiography was performed on 42 patients with acute chest pain to explore the value of 64-row spiral CT cardiothoracic combined angiography in the diagnosis of the cause of acute chest pain.

## 2. Data and Methods

### 2.1. Research Subjects

There were 27 male and 15 female cases. The mean age of the patients was 61.5 years, ranging from 38 to 81 years. All patients had no significant abnormalities on electrocardiogram before the combined cardiothoracic angiography, and their past medical history did not accurately suggest the cause of acute chest pain. Patients with contrast allergy, severe renal insufficiency, and severe arrhythmias were excluded from this study. Selective coronary angiography was performed within 1 week of admission in 6 patients with coronary artery stenosis (see Table 1).

RETRACTED

### 2.2. Research Methods

The patient was scanned in the supine position, from the thoracic inlet to the base of the heart, in the cephalic direction. Scanning parameters: collimation width 0.625 mm, pitch 0.2, effective layer thickness 0.8 mm, recombination interval 0.4 mm, tube voltage 120 kV, tube current 400 mA, and tube rotation time 0.4 s. A double-barrel high-pressure syringe was used, and the nonionic contrast agent Uvexan (370 mgI/ml) 100 ml was used. The contrast medium was injected from the left elbow vein at a flow rate of 5.0 ml/s (80 ml), followed by 20 ml of contrast medium at a flow rate of 3.0 ml/s and 40 ml of physiological saline at the same flow rate, and was monitored at the level of the descending aorta near the main pulmonary artery using an intelligent trigger scan. The trigger threshold was 120 HU, and the scan delay time was 5 s.

The coronary artery was reconstructed first by retrospective ECG gating technique, and the end-diastolic phase (i.e., 75% of the RR interval) was reconstructed because the heart beat was weak in this phase, which had the least impact on the quality of the reconstructed images. If the image quality was not satisfactory, the original data were reconstructed at 5% intervals between 20% and 80% of the RR interval, and the R-R interval with the best image quality was selected for coronary image reconstruction. Stenosis was assessed according to the American Heart Association 15-segment coronary artery segmentation method, and the criteria for stenosis were mild stenosis of ≤50%, moderate stenosis of 51% to 75%, and severe stenosis of ≥76%. In all patients, multiplanar reconstruction (MPR), curved planar reconstruction (CPR), volume rendering (VR), and maximal density projection (MDP) were performed. For the lesioned vessels, the 3D reconstructed images were analyzed together with the original cross-sectional images, and the area of interest was viewed from multiple angles to best show the lesion. All patients were diagnosed independently by two experienced radiologists, and in case of disagreement, the final conclusion was made by a chief physician.

### 2.3. Statistical Processing

The data were statistically processed using SPSS22.0 software, and the count data were expressed as rate by *χ*2 test; the measurement data of normal distribution were expressed as *x* ± *s*, in which the *t*-test was used for the paired control group within the group and the *t*-test for two independent samples between the groups; and the measurement data of nonnormal distribution were tested by rank sum test, and the difference was considered statistically significant at *P* < 0.05.

## 3. Diagnosis of Acute Chest Pain

### 3.1. Acute Coronary Syndrome

Acute coronary syndromes are a group of clinical syndromes caused by coronary atherosclerotic plaque invasion candling or rupture or vascular epidural contracture, resulting in the formation of complete or incomplete occlusive thrombus, leading to acute or subacute myocardial ischemia. The syndrome includes unstable angina pectoris, acute nonsegment elevation myocardial infarction, acute segment elevation myocardial infarction, and sudden ischemic cardiac death. Unstable angina and nonsegment elevation myocardial infarction often result in partial or intermittent obstruction of the coronary lumen, while segment elevation myocardial infarction often results in coronary artery obstruction. Acute coronary syndrome is a common and serious life-threatening cardiovascular disease. Acute coronary syndromes arise from the rupture of atherosclerotic plaques in the coronary arteries, accompanied by platelet aggregation and thrombosis.

RETRACTED

In the past, it was thought that the pathogenesis was caused by the thickening of the atheromatous plaque causing luminal narrowing, which leads to insufficient blood supply from the coronary arteries to the myocardium. The clinical symptoms of the acute coronary syndrome are related to the degree of coronary artery obstruction, as shown in Figure 2. The most typical clinical symptom is angina pectoris. In patients with unstable angina, the symptoms of chest pain often occur with mild exercise or at rest. In patients with nonsegment elevation myocardial infarction, chest pain is longer and more severe than in unstable angina. The typical manifestation of angina is episodes of retrosternal dullness or pressure or burning sensation, which may be accompanied by ulnar radiating pain to the left upper arm, left jaw, left neck, left back or shoulder, and left forearm, either intermittently or continuously. Some patients may have sweating, dyspnea, nausea, or even syncope, which can last from up to minutes and often indicates acute myocardial infarction if it is not completely relieved with glycerol. Atypical manifestations include toothache, epigastric vague pain, sore throat, pins and needles pain in the chest, and dyspepsia. Acute coronary syndrome is a serious life-threatening condition that can lead to heart failure and arrhythmias. Early diagnosis can reduce the death rate and improve the prognosis of patients.

### 3.2. Pulmonary Artery Embolism

Pulmonary embolism is a group of clinical syndromes caused by the obstruction of the pulmonary artery and its branches by emboli of various components. The most common source of emboli can be emboli in the venous system of the body circulation; embolism can also be fat embolism, amniotic fluid embolism, and air embolism. The emboli obstruct the pulmonary arteries or their branches, causing a reduction or interruption of blood flow to the corresponding blood supplying lung tissue and necrosis of the lung tissue in the area of blood supply. Among the various sources of emboli, lower extremity deep vein thrombosis is the most common. In proximal lower extremity deep vein thrombosis, approximately patients will present with symptoms of pulmonary embolism, while in patients with pulmonary embolism, if a sensitive diagnostic method is used, some patients will be found to have lower extremity deep vein thrombosis. Pulmonary embolism is often fragmented and can be easily misdiagnosed and missed clinically. Studies have shown that the mortality rate of acute pulmonary embolism in patients with pulmonary embolism is due to failure in treatment, and the mortality rate of patients with pulmonary embolism who are treated is low; therefore, early diagnosis of pulmonary embolism is critical. The clinical manifestations of pulmonary embolism are varied and lack specificity, as shown in Figure 3. Early atypical clinical manifestations include fever, cough, transient shortness of breath, palpitations, and decreased blood pressure. Typical patients with pulmonary embolism may present with sudden dyspnea, chest pain often aggravated by inspiration, hemoptysis, and a violent cough.

RETRACTED

Although 64-row spiral CT combined cardiothoracic angiography can clearly display the thoracic aorta, both pulmonary arteries, coronary arteries and their major branches, several problems are faced during the scanning process: (1) breath-holding time: coronary artery imaging requires very high breath-holding, and the scanning range of combined cardiothoracic imaging is from the lung tip to the diaphragm including the whole lung field, which is significantly larger than the traditional coronary CTA scanning range. The combined cardiothoracic imaging scan range is significantly larger than the conventional coronary CTA scan range, and a scan time of 16 to 18 s is difficult for patients with acute chest pain to cooperate. (2) Heart rate: in this scan, retrospective ECG gating is used, so the heart rate also affects the image quality, and most patients with emergency chest pain have a fast heart rate. (3) Radiation dose: 64-row spiral CT cardiothoracic combined angiography uses a thin layer and small pitch scanning, and the radiation dose to patients is significantly higher.  Figure 4 shows the relationship between radiation dose and imaging quality. Therefore, how to minimize the radiation dose has become a hot issue nowadays while ensuring the quality of the scan. It has been found that prospective cardiac gating reduces the effective radiation dose by an average of 60% compared to retrospective cardiac gating without compromising image quality, which is a trend toward continuous improvement of combined cardiothoracic angiography protocols.

RETRACTED

### 3.3. Aortic Coarctation

Aortic coarctation accounts for approximately the proportion of acute aortic syndromes. Aortic coarctation is an entrapment hematoma formed when blood circulating within the aorta enters the middle layer of the aorta from a torn intimal rupture, and the hematoma divides the aorta into a true lumen and a false lumen. The mortality rate of aortic coarctation is high and it is one of the most critical diseases in cardiovascular disease. Early diagnosis and reasonable and active treatment are the keys to reduce the mortality rate. The main symptom of the entrapment is a sudden onset of severe tearing pain with very characteristic manifestations, and the pain can migrate downward. The site of pain often correlates with the location of the rupture tear, such as anterior pain located in the chest, suggesting that the tear may be located in the ascending aorta, while back pain is closely related to descending aortic entrapment. The main types of aortic coarctation in typing are type and type, which are based on whether the ascending aorta is involved. Type is aortic coarctation involving the ascending aorta or aortic arch. The endothelial rupture is located in the ascending aorta or aortic arch. The type of aortic coarctation involves the descending aorta, but not the ascending aorta or aortic arch. There are three main types: type 1 rupture is located in the ascending aorta and the entrapment involves the aortic arch; type 2 rupture is located in the ascending aorta and the entrapment involves only the ascending aorta; type 3 rupture is located in the descending aorta and the entrapment involves the distal part of the aorta. The treatment of aortic coarctation is related to the staging of the coarctation. For type 2 clips, surgical treatment is more effective than pharmacological treatment, as shown in Figure 5. In contrast, for type 2 clips without comorbidities, the effect of pharmacological treatment was better than that of surgical treatment.

In patients with acute coronary syndrome, the diagnosis of segmental elevation myocardial infarction can generally be made based on the patient′s symptoms, signs, chest radiograph, electrocardiogram, and laboratory findings including myocardial enzymology, and other conditions are divided into three categories: the first category is acute coronary syndrome high-risk group or nonsegmental elevation myocardial infarction, the second category is acute coronary syndrome low-risk group, and the third category is noncardiogenic chest pain. The more commonly used clinical risk score is the Infarct Thrombosis Risk Score, which predicts whether a new infarction, old infarction, or the need for revascularization within a week will be assessed in the following areas: age greater than or equal to years, history of coronary artery disease (documented coronary stenosis greater than or equal to three risk factors for cardiovascular disease (age, male family history, diabetes, hyperlipidemia, smoking, and obesity), aspirin use within the last days, ECG segmental changes (persistent decrease or transient elevation), increased myocardial enzymes, and angina symptoms more than twice within an hour.

RETRACTED

Each of the above assessments is scored, and if the score is a score or points, then it is a low-risk group. Patients who are in the high-risk group for acute coronary syndrome or nonsegment elevation myocardial infarction usually require hospital admission. Patients with noncardiogenic chest pain of nonfatal etiology usually require follow-up only. Patients in the low-intermediate risk group for acute coronary syndrome usually require a period of observation and a series of myocardial enzymatic tests, and hospitalization if myocardial enzymatic results are elevated. For patients in the low-intermediate risk group for acute coronary syndrome, there will still be a proportion of patients requiring hospitalization who will be treated as a follow-up, which can significantly increase patient mortality. In patients with nonsegmental alterations of infarction, the cost of screening can be reduced if accurate predictors of high-risk factors are available or if coronary syndromes can be excluded earlier during the observation period. In addition, early identification of patients in the high-risk group for acute coronary syndromes allows for early treatment. Cui et al. provide a rational recommendation for the examination process for patients with suspected myocardial ischemia: based on the patient′s symptoms, signs, chest radiograph, electrocardiogram, and whether laboratory tests including myocardial enzymology can diagnose segmental elevation myocardial infarction, nonsegmental elevation myocardial infarction, and nonspecific changes; for the first two, the patient needs to be admitted to the hospital, and if the coronary findings in nonspecific patients show that stenosis is greater than 50%, admission is required, and if the stenosis is less than 50%, no hospitalization is required, and if it is equal to 50%, additional testing is required to confirm the diagnosis.

RETRACTED

## 4. Results and Discussion

The 64-slice spiral CT combined cardiothoracic angiogram of 42 patients clearly showed the thoracic aorta, both pulmonary arteries, the main coronary arteries and their major branches (see Figure 6), of which 18 patients showed a total of 27 coronary arteries with varying degrees of stenosis. A total of 11 coronary arteries were found to have stenosis greater than 50% in 6 patients with coronary artery stenosis. After admission, selective coronary angiography was performed, and the results were all consistent with CT combined cardiothoracic angiography. Seven cases of aortic coarctation were classified according to Debakey′s classification, two cases of type I and five cases of type III. Acute pulmonary artery embolism was diagnosed in 6 cases, including 4 cases above the segment and 2 cases below the segment. Pneumothorax was also diagnosed in 4 cases, and no significant abnormalities were seen in 7 cases.

The sensitivity of 64-row spiral CT coronary imaging in the diagnosis of coronary artery stenosis ≥50% was 93%, the specificity was 98%, and the average negative predictive value was 97%. The ability of MSCT coronary imaging to quantitatively assess the severity of coronary artery disease has also been studied, and it has been found to correlate well with coronary angiography, making it a valuable clinical tool for the detection and exclusion of coronary artery disease. 64-row spiral CT combined cardiothoracic angiography uses a retrospective cardiac gating technique to obtain the optimal contrast in a single scan. The cross-sectional images of the thoracic arteries in the filling state are obtained in one scan, and then the thoracic aorta, both pulmonary arteries, coronary arteries and their major branches are reconstructed by different postprocessing methods such as MPR, MIP, CPR, and VR. All 42 patients in this group showed the above vessels clearly in one scan, as shown in Figure 7, and made a correct diagnosis of their diseases. The main symptom of the entrapment is a sudden onset of severe tearing pain with very characteristic manifestations, and the pain can migrate downward. The site of pain often correlates with the location of the rupture tear, such as anterior pain located in the chest, suggesting that the tear may be located in the ascending aorta, while back pain is closely related to descending aortic entrapment. There are two main types of aortic staging: staging and staging. The main types of aortic coarctation in typing are type and type, which are based on whether the ascending aorta is involved. Type is aortic coarctation involving the ascending aorta or aortic arch. The endothelial rupture is located in the ascending aorta or aortic arch. The type of aortic coarctation involves the descending aorta, but not the ascending aorta or aortic arch.

RETRACTED

For patients with acute chest pain, after taking a medical history, emergency physicians usually perform ECG, cardiac ultrasound (USG), etc. For patients considering acute myocardial infarction, they also perform myocardial radionuclide imaging and serum marker testing. Sometimes, the treatment time of critical patients with acute chest pain is delayed, and each test can only make a direct or indirect diagnosis of a certain disease. Cardiac ultrasound can detect thoracic aortic coarctation, but the rupture of the aortic coarctation is not clearly shown, and the diagnosis of acute myocardial infarction can only be made indirectly by the movement of the myocardium. DSA is the gold standard for the diagnosis of vascular diseases, but it is an invasive test, and DSA cannot show coronary artery, pulmonary artery, and thoracic aorta at the same time, so it cannot diagnose nonvascular diseases. 64-slice CT combined cardiothoracic angiography can not only make the correct diagnosis of vascular diseases in the chest but also accurately understand the condition of both lung tissues, mediastinum and pericardium. 64-slice CT combined cardiothoracic angiography requires simultaneous imaging of the thoracic aorta, both pulmonary arteries, coronary arteries and their major branches. This poses a challenge in terms of timing, scan start time, and contrast dosage because the peak of pulmonary artery enhancement (9–12 s) is earlier than that of the aorta and coronary artery (16–22 s), as shown in Figure 8, so that clear images of the coronary artery, pulmonary artery, and aorta are obtained simultaneously. Therefore, to obtain clear images of the coronary artery, pulmonary artery, and aorta at the same time, it is crucial to extend the enhancement time of the pulmonary artery.

There are several options for the use of contrast agents:

1. Increase the total amount of contrast agent: the total amount of contrast agent was obtained by calculating the formula ((right pulmonary artery peak time–aortic peak time) + scan length) × injection rate (5 ml/s), which was 135 ml on average. However, the total amount of contrast agent was still high (137 ml on average).
2. Biphasic injection: a biphasic injection scheme can be used to obtain uniform and obvious intensification of the three major vessels, i.e., high flow rate of 5 ml/s and flow rate of 100 ml in phase 1, reduced flow rate of 3 ml/s and flow rate of 30 ml in phase 2, and total 130 ml of contrast agent.
3. Three-phase injection: the first two phases were injected with the same amount of contrast agent as the two phases, and the third phase was injected with 30–50 ml of saline. Then, we injected 40 ml of physiological saline at the same flow rate and obtained very satisfactory results.

RETRACTED

We found that this scheme resulted in less flow artifacts in the right ventricle and more uniform right ventricular enhancement, which avoided compromising the image quality of the right coronary artery, and that we used a foot-head orientation to obtain early images of distal pulmonary artery enhancement at the base of the lung.

## 5. Conclusion

In this paper, we focus on the value of 64-row spiral CT cardiothoracic combined angiography in acute chest pain. The results show that 64-row spiral CT has the advantages of fast scanning speed, high resolution, and advanced postprocessing technology, and combined cardiothoracic angiography can quickly and accurately help emergency physicians analyze the cause of acute chest pain, which plays a very important role in formulating the correct treatment plan in a timely manner. The main symptom of the entrapment is a sudden onset of severe tearing pain with very characteristic manifestations, and the pain can migrate downward. The site of pain often correlates with the location of the rupture tear, such as anterior pain located in the chest, suggesting that the tear may be located in the ascending aorta, while back pain is closely related to descending aortic entrapment. At the same time, with the continuous development of CT technology, the temporal and spatial resolution has improved the quality of CT images, giving us more options to reduce the effective radiation dose and reduce the total amount of contrast, making the 64-row spiral CT cardiothoracic imaging more perfect.

## Figures and Tables

**Figure 1:** One-stop imaging for chest pain triad.

**Figure 2:** Acute coronary pathogenesis.

**Figure 3:** Changes in venous CTQ protein index during the pathogenesis of pulmonary embolism.

**Figure 4:** Relationship between radiation dose and imaging quality of 64-row spiral CT cardiothoracic combined angiography.

**Figure 5:** Comparison of the effect of surgical treatment with that of drug treatment.

**Figure 6:** 64-row spiral CT combined cardiothoracic angiography.

**Figure 7:** Cross-sectional image index changes of thoracic arteries.

**Figure 8:** Peak pulmonary artery enhancement.

**Table 1:** The general information of selected patients.

Group	Average age (weeks)	Gender (male/female)	Disease duration (month)	Injury part	
				Arterial narrowing	Arteriosclerosis
Control	38–81	27/15	0.83 ± 0.12	6	36
Observation	38–81	24/18	0.76 ± 0.07	9	33

## Data Availability

The data used to support the findings of this study are available from the corresponding author upon request.
